RETRACTED

# Analysis of Adverse Pregnancy Outcomes of Pregnant Women with Syphilis and Maternal-Infant Serological Association in Changzhou, China, 2015–2019

**DOI:** 10.1155/2022/9673850

**Published:** 2022-09-05

**Authors:** Chaorong Bian, Zhiqiang Qin, Jieying Zhang, Mengtao Sun, Manman Gu, Kejin Chen

**Affiliations:** ^1^Changzhou Children's Hospital Affiliated to Nantong University, Changzhou, 226019 Jiangsu, China; ^2^Changzhou Maternal and Child Health Care Hospital, Changzhou Medical Center, Nanjing Medical University, Changzhou, 213000 Jiangsu, China; ^3^Department of Epidemiology and Biostatistics, School of Public Health, Medical College of Soochow University, Suzhou, 215123 Jiangsu, China

## Abstract

**Background:**

Although the prevention of mother-to-child transmission of syphilis program in China has achieved national coverage for 7 years, controversy still exists regarding the treatment of syphilis and the serological significance of syphilis.

**Objective:**

To explore the occurrence and influencing factors of adverse pregnancy outcomes among pregnant women with syphilis in Changzhou from 2015-2019 and to further analyze the impact of syphilis serologic titers on perinatal outcomes and neonatal serologic outcomes.

**Methods:**

Syphilis-infected pregnant women reported in Changzhou City from 2015 to 2019 were selected as the study population (data were obtained from the “China Information System for Prevention of Mother-to-child Transmission of AIDS, Syphilis and Hepatitis B.” Demographic characteristics, laboratory tests, and medication were collected to describe adverse pregnancy outcomes and the distribution of non-pale leptospiral antibody titers during pregnancy. Multivariate logistic regression was used to analyze the factors influencing adverse pregnancy outcomes. We also compared differences in syphilis titers among mothers who received different interventions, differences in serologic outcomes of their children, and correlations between them.

**Results:**

For mothers with syphilis infection, we found no treatment during pregnancy (OR =1.70) and an initial titer greater than 1 : 8 (OR =2.28) to be risk factors. For treated pregnant women, increasing age (OR =1.08), lack of standardized treatment (OR =1.87), and initial titer greater than 1 : 8 (OR =1.69) were risk factors, while previous parity was a protective factor (OR =0.62). For untreated pregnant women, marital status (OR =2.40) and initial titers greater than 1 : 8 (OR =3.57) were risk factors. There were statistically significant differences (*P* < 0.01) in serologic titer changes, time to antibody regression, and time to exclusion of syphilis infection in children of pregnant women with syphilis infection after receiving different interventions during pregnancy, but different time distributions of interventions had no effect on these three indicators.

RETRACTED

**Conclusion:**

Pregnant women with syphilis should actively cooperate with their doctors in the standardized treatment of pregnancy, and doctors should also pay more attention to pregnant women with syphilis whose initial titers are greater than 1 : 8. High-quality prenatal care is a key component in interrupting mother-to-child transmission of syphilis and preventing various adverse pregnancy outcomes. The adaptation of standardized treatment protocols for pregnant women with syphilis in China is a strong proof of the progress of precision medicine.

## 1. Introduction

Syphilis infection in pregnancy has been on the rise in recent years, and there have been more clinical investigations of pregnancy outcomes in syphilis infection in pregnancy, and some data [1, 2] show that adverse pregnancy outcomes are significantly higher in patients with syphilis during pregnancy than those in normal pregnancies. The more common adverse pregnancy outcomes in patients with syphilis in pregnancy include miscarriage, preterm delivery, stillbirth, intrauterine distress, low birth weight babies, and congenital syphilis in newborns [3, 4]. Combined syphilis infection in pregnancy is a high-risk pregnancy and is an unfavorable factor for maternal and infant safety.

Standardized treatment is an indispensable stage to achieve mother-to-child interruption in pregnant women infected with syphilis. However, after treatment, some women's non-pallidoglobulin antibody titers fall to a certain level (usually ≤1 : 8) and then stop falling. The titer will remain stable at a low level for a long time, even for life, as a serological fixation phenomenon [5]. Since it is unclear whether this phenomenon indicates persistent infection in patients or represents a sustained autoimmune response induced by the infection, there is still controversy as to whether and how to treat the serologically fixed syphilis population [6].

Some studies have shown that the titer of non-pale spirochete antibodies is less related to the duration of the disease and more to the body's response to pale spirochetes [7]. A key issue in evaluating efficacy with titers is the extent to which titers reflect the true disease activity of syphilis. Whether high and low titers are consistent in reflecting the activity status of pallidospiral infection and whether there are differences in serologic findings in neonatal syphilis are possible research gaps.

Currently, most national studies have only investigated the relationship between treatment during pregnancy and pregnancy outcome in pregnant women with syphilis infection [8–11], and few studies have evaluated the relationship between their treatment during pregnancy and the conversion of syphilis-specific antibodies in those children exposed to syphilis. It is worth mentioning that the change in serological titers before and after treatment was not identical in each pregnant woman with syphilis infection. In conclusion, the aim of this study was to examine the impact of changes in nonspecific antibody titers in syphilis-infected pregnant women on perinatal outcomes and serology to provide an accurate basis for the development of comprehensive interventions to prevent mother-to-child transmission of syphilis (MTCT).

RETRACTED

## 2. Materials and Methods

### 2.1. Study Population

Inclusion criteria: Pregnant women with positive results of Treponema pallidum serological test and non-Treponema pallidum antigen serological test, and the gestational age ≥28 weeks. Exclusion criteria: The reporting conditions are not met due to the lack of important personal information and other reasons.

### 2.2. Testing Method

Syphilis serological detection methods include non-Treponema pallidum antigen serological test and Treponema pallidum antigen serological test. The non-Treponema pallidum serological test uses the rapid plasma reagin ring card test (RPR, InTec®). Treponema pallidum serological test adopts Treponema pallidum particle agglutination test (TPPA, Autobio®).

### 2.3. Treatment Plan

The standard treatment of syphilis-infected pregnant women must meet the following conditions at the same time (2015 version) [12]: the application of adequate penicillin treatment; two courses of treatment during pregnancy, with an interval of more than 2 weeks between the two courses; the second course of treatment is carried out and completed in the third trimester of pregnancy.

The neonatal treatment plan is to apply benzathine penicillin G 50,000 U/kg after birth, 1 intramuscular injection, divided into the gluteal muscles on both sides.

### 2.4. Outcome Indicators

Adverse pregnancy outcomes include stillbirth, death within 7 days, prematurity or low birth weight, birth defects, neonatal pneumonia, neonatal asphyxia, and neonatal congenital syphilis.

Children exposed to syphilis are followed up at 3, 6, 9, 12, 15, and 18 months after birth, including child care and associated serologic testing for syphilis. Children born to syphilis-infected pregnant women were followed up to 21 months old and the infection status could not be determined, which was defined as loss to follow-up. Syphilis infection can be ruled out if all the non-Treponema pallidum antigen serological tests at 0, 3, and 6 months old are negative for infants born to syphilis-infected mothers, or if any TPPA test is negative within 18 months old.

RETRACTED

### 2.5. Statistical Analysis

All data are from China Information System for Prevention of Mother-to-Child Transmission of Syphilis. The system has been used to monitor and assess the prevalence of maternal syphilis and congenital syphilis in China.

Excel 2010 was used to organize and check the data, and R (4.0.2) was used for statistical analysis. The age of the study subjects conformed to a normal distribution and was expressed as $\bar{x}\pm s$. The *χ*^2^ test was used to compare the incidence of adverse pregnancy outcomes in subjects with different characteristics. An unconditional multivariate logistic regression model was constructed to analyze the factors associated with adverse pregnancy outcomes. The relationship between maternal RPR titers and neonates was analyzed bivariate using the Spearman rank correlation test and two independent samples using the Wilcoxon rank sum test. *P* < 0.05 was considered statistically significant.

## 3. Results

The average age of the 489 subjects was 29.13 ±5.42 years old, and most of them were 25-29 years old, accounting for 40.29% (197 cases). The majority were Han nationality, accounting for 96.32% (471 cases), and most of their education level were junior high school and high school, accounting for 57.67% (282 cases) (Table 1).

Among the 489 subjects, 311 (63.6%) were treated for syphilis. And 136 (43.73%) of the 311 subjects received the standardized treatment. There were 164 cases of adverse pregnancy outcomes, and the overall incidence was 33.54%. The incidences in treated and untreated patients were 29.90% (93/311) and 39.89% (71/178), respectively, and there was a statistically significant difference (*P* = 0.025). The incidence of adverse pregnancy outcomes in standardized treatment and non-standardized treatment was 23.53% (32/136) and 34.86% (61/175), respectively, with a statistically significant difference (*P* = 0.030) (Table 1).

There were no statistically significant differences in the incidence of adverse pregnancy outcomes among the subjects of different age groups (*P* = 0.460). The differences of the incidences of adverse pregnancy outcomes in different period of diagnosis of syphilis infection were statistically significant (*P* = 0.032). The highest incidence was 50% (14/28) in the group of diagnosed as syphilis after delivery and the lowest was 31.37% (133/424) in the group of diagnosed during pregnancy (Table 1).

We used the adverse pregnancy outcome as the dependent variable and took most general information of all the subjects as the independent variables. All variables were included in an unconditional multivariate logistic regression model (Model 1, Hosmer Lemeshow Test, *χ*^2^ = 14.882, df = 7, *P* = 0.038) to analyze the factors associated with adverse pregnancy outcomes. Those with titers greater than or equal to 1: 8 were more likely to have adverse pregnancy outcomes compared with those with titers less than 1: 8 at the initial test (OR =2.282, 95% CI, 1.435-3.361). Compared with the untreated mothers, the treated were less likely to have adverse pregnancy outcomes (OR = 0.588, 95% CI, 0.394-0.877) (Table 2).

RETRACTED

In this study, to further analyze the impact of standardized treatment on adverse pregnancy outcomes, we took the treated pregnant women as the research object. And receiving the standardized treatment or non-standardized treatment was included as independent variable in the logistic regression model (Model 2, Hosmer Lemeshow Test, *χ*^2^ = 6.461, df = 8, *P* = 0.596) under the condition that other independent variables remained unchanged. The risk of adverse pregnancy outcomes increased by 7.9% for each year of maternal age with syphilis infection (1.079, 95% CI, 1.026-1.134). For women with syphilis infection, the risk of adverse pregnancy may decrease by 37.6% for each grade of previous parity (OR =0.624, 95% CI, 0.416-0.937). The results showed that compared with the non-standardized treatment for syphilis, the standardized treatment was less likely to have adverse pregnancy outcomes (OR = 0.534, 95% CI, 0.314-0.906) (Table 3).

We also took the untreated pregnant women as the research object and constructed the logistic regression model (Model 3, Hosmer Lemeshow Test, *χ*^2^ = 1.558, df = 2, *P* = 0.459). Those with other marital statuses were more likely to have adverse pregnancy outcomes compared with those who were first married (OR = 2.395, 95% CI, 1.041-5.508). Those with titers greater than or equal to 1: 8 were more likely to have adverse pregnancy outcomes compared with those with titers less than 1: 8 at the initial test (OR = 3.568, 95% CI, 1.348-9.442) (Table 4).

There was a statistically significant difference in the changes in serological titers (initial titers minus prepartum titers) among syphilis-infected pregnant women after receiving no treatment, one or two courses of treatment during pregnancy (*P* < 0.01). For the children born to the three groups of pregnant women, the difference in the months when their syphilis-specific antibodies turned negative was statistically significant (*P* = 0.01), and the difference in the months when syphilis infection was excluded was also statistically significant (*P* = 0.01) (Table 5).

RETRACTED

For pregnant women with syphilis who received only one course of treatment, the treatment time was in the first trimester, second trimester, and third trimester, respectively, and there was no significant difference in serological titers (*P* = 0.06). There was no statistical significance in the time of antibody conversion and exclusion of syphilis infection in their children (Table 6).

Similarly, after receiving 2 courses of treatment, although the treatment time distribution was different, the three indicators were not statistically significant (Table 7).

For pregnant women with syphilis that were serologically fixed, that is, they did not receive treatment, received one or two courses of treatment with no change in serological titers during pregnancy, there was no statistically significant difference in the time of antibody conversion and exclusion of syphilis infection in their children (Table 8).

The high titer group (≥1 : 32) and the low titer group (≤1 : 8) received no treatment, one or two courses of treatment during pregnancy, the differences in serological titers were statistically significant (*P* < 0.01), but there was no statistically significant difference in the metastasis and development of serology among the children (Table 9).

## 4. Discussion

This study showed that the incidence of adverse pregnancy outcomes among syphilis-infected pregnant women in Changzhou City, Jiangsu Province, was 33.54% from 2015 to 2019, which was significantly higher than the 12.0% previously reported in Jiangsu Province from 2013 to 2016 [8]. On the one hand, more pregnant women with occult syphilis are tracked due to the improvement of information technology; on the other hand, Changzhou is an economically developed area with a high proportion of mobile infected pregnant women, making intervention difficult. Carles G [13] conducted a retrospective study in France to assess the effects of syphilis in pregnancy on the fetus and newborn, suggesting an overall incidence of adverse pregnancy outcomes of 34.1%, which is similar to our study. Although the population composition, stage of disease, and definition of indicators may vary between countries, the results suggest that pregnant women with syphilis are equally at high risk of adverse pregnancy outcomes.

In our retrospective study, among untreated mothers with syphilis, the incidence of adverse pregnancy outcomes was 39.89%, lower than the pooled estimate of 76.8% for all APOs reported in the previous meta-analysis [14]. In the future, it is particularly important to explore individualized intervention models suitable for these underserved populations and to strengthen informatization construction.

RETRACTED

Our team found that a higher proportion of infected pregnant women across the city were less educated, homemakers, and jobless women. This group is often disadvantaged in terms of family status and lack of self-care awareness, which affects the timeliness of detection and treatment. The knowledge and skills of the first-visit obstetricians and gynecologists in grassroots medical institutions, IPMTCT service awareness, and familiarity with relevant national policies, as well as whether to provide health education for the target population, will become the key links to increase the proportion of pregnancy testing in the future. In addition, pregnant women's awareness of IPMTCT-related knowledge also affects their willingness and behavior to receive early detection [15]. Therefore, comprehensive community support and care activities should be carried out, and more effective publicity and mobilization models should be explored.

We studied the incidence of adverse pregnancy outcomes and found that there were differences in the period of diagnosis, gestational weeks at diagnosis, initial test titer, whether to treatment, and whether to standardized treatment. Based on these univariate analysis results and relevant professional knowledge, and then including all the corresponding independent variables, we constructed regression models 1, 2, and 3, respectively.

For syphilis-infected mothers, we found that no treatment during pregnancy and initial titer greater than 1 : 8 were risk factors. Pregnancy syphilis is mainly latent syphilis, and the infection symptoms are not obvious. Therefore, regular monitoring of non-Treponema pallidum antibody titers for pregnant women infected with syphilis is of great significance for judging the treatment effect and diagnosis of neonatal congenital syphilis [16]. The higher the titer during pregnancy, the higher the risk of adverse pregnancy outcomes such as miscarriage, preterm birth, stillbirth, and congenital syphilis [17, 18].

Taking the treated and non-treated pregnant women as a separate group, respectively, we have found new concerns. For pregnant women receiving treatment, increasing age, lack of standardized treatment, and initial titer greater than 1 : 8 are risk factors, while parity is a protective factor. From Table 1, it is clear that the results of the group over the age of 35 have an impact on the overall, and for all pregnant women over the age of 35, all body functions will decline, and the probability of various pregnancy syndromes and fetal malformations will also increase [19]. Standard treatment is more effective than non-standard treatment, and the key may lie in two courses of treatment. On the one hand, the treatment time is long, and it plays a blocking role in the most likely occurrence of fetal syphilis. On the other hand, if the drug did not work in the first course of treatment, those pregnant women could have a second course of treatment as a complementary treatment. Regardless of PMTCT is successful after treatment before first delivery, or the untreated may result in adverse pregnancy outcomes in first delivery, both may lead to more pregnant women taking the initiative to join the team for treatment in subsequent deliveries.

RETRACTED

However, if the target population was untreated pregnant women, the results were different, with marital status and primary titers greater than 1 : 8 being risk factors. Marital satisfaction was higher in first marriages than in remarriages and divorces, which had an impact on fertility [20]. Pregnant women in first marriages and their partners are more concerned about their children and more willing to be treated for syphilis.

If these mothers receive treatment during pregnancy, the time for the children to rule out syphilis infection or turn negative for antibody will be shorter; otherwise, the time will be longer, and even congenital syphilis may be finally diagnosed [21, 22]. But whether it is one course or two courses, the time distribution of receiving treatment can be different, because our study shows that when the mothers are treated does not affect the children's serological status. Pregnant women with syphilis serofixation, whether treated or not, had no effect on children's outcomes, probably because Treponema pallidum had been cleared from the body at this time, showing persistently positive titers, but how to define serological fixation still lacks a clear standard, so treatment is still necessary. Although the changes in titers were inconsistent between the high titer group and the low titer group after receiving the same intervention, the outcomes of children were consistent, which also meant that the high titer group did not require more courses of treatment. At the end of 2020, the National Health Commission of China optimized the standard treatment plan for PMTCT of syphilis, deleted the original “required two courses of treatment,” and “the second course of treatment is carried out and completed in the third trimester” was changed to “treatment should be completed one month before delivery” [12, 23]. These findings of our study may also shed light on the reasons for the optimization scheme.

## 5. Limitations

This study has some limitations. The data used in this study are the registration data of the national routine work information system, and there is a lack of specific collection and analysis of risk factors for some adverse pregnancy outcomes. Moreover, the data are not primary clinical data, and there may be information bias in the retrospective data of treatment and laboratory tests. In addition, the included research subjects were syphilis pregnant women who gave birth after 28 weeks, and the miscarriage in the first and second trimesters was not considered, which may underestimate the occurrence of adverse pregnancy outcomes in syphilis-infected women.

RETRACTED

## 6. Conclusions

In summary, pregnant women with syphilis should keep the serological titer below 1 : 8 before pregnancy and actively cooperate with doctors to do standard treatment during pregnancy, which can effectively prevent the occurrence of adverse pregnancy outcomes and can also make the syphilis-specific antibodies of their children turning negative as soon as possible to rule out syphilis infection. It is necessary to establish an innovative working model that protects privacy and allows pregnant women and their sexual partners to receive standardized anti-syphilis treatment at the same time, thereby effectively reducing the positive rate of neonatal serological syphilis testing and the incidence of congenital syphilis. The key to the success of the program to prevent and control MTCT of syphilis lies in the early diagnosis, early treatment, and standardized follow-up of syphilis-positive pregnant women [24]. A region can rely on the sexually transmitted disease (STD) epidemic monitoring network to form a referral pattern centered on treatment and follow-up institutions, and at the same time use government actions to supervise and evaluate related work, fundamentally improving the quality of project operation.

## Figures and Tables

**Table 1:** General information of the research objects and comparison of the incidence of adverse pregnancy outcomes.

General information	Number of research objects	Constituent ratio (%)	Adverse pregnancy outcomes			
			Number of cases	Incidence (%)	*χ* ^2^	*P*
Age					2.59	0.46
<25	91	18.61	30	32.97	—	—
25~	197	40.29	64	32.49	—	—
30~	115	23.52	35	30.43	—	—
>=35	86	17.59	35	40.70	—	—
Nationality					0.63	0.426
Han nationality	471	96.32	157	33.33	—	—
The other	18	3.68	7	38.89	—	—
Degree of education					3.43	0.488
Primary school and below	40	8.18	16	40.00	—	—
Junior high school	148	30.27	50	33.78	—	—
High school	134	27.4	50	37.31	—	—
College/university	111	22.7	31	27.93	—	—
Unknown	56	11.45	17	30.36	—	—
Occupation					8.32	0.139
Worker	84	17.18	31	36.90	—	—
Farmer	27	5.52	5	18.52	—	—
Business	49	10.02	15	30.61	—	—
Professional skill worker	13	2.66	3	23.08	—	—
Housework or unemployed	234	47.85	74	31.62	—	—
The other	82	16.77	36	43.90	—	—
Marital status					3.63	0.057
First marriage	396	80.98	125	31.57	—	—
The other	93	19.02	39	41.94	—	—
Previous infection					0.97	0.324
Yes	212	43.35	66	31.13	—	—
No	277	56.65	98	35.38	—	—
Diagnosis period					6.86	0.032
Pregnancy	424	86.91	133	31.37	—	—
During childbirth	37	7.57	17	45.95	—	—
After delivery	28	5.52	14	50.00	—	—
Weeks of first antenatal visit					0.80	0.849
<13	321	65.64	106	33.02	—	—
13-	116	23.72	39	33.62	—	—
>=28	46	9.41	16	34.78	—	—
Unknown	6	1.23	3	50.00	—	—
Weeks of diagnosis of syphilis infection					6.54	0.038
<13	126	25.77	33	26.19	—	—
13-	155	31.70	49	31.61	—	—
>=28	208	42.54	82	39.42	—	—
Titers of first antenatal visit					7.88	0.005
<8	382	78.12	116	30.37	—	—
>=8	107	21.88	48	44.86	—	—
Syphilis treatment					5.06	0.025
Yes	311	63.6	93	29.90	—	—
No	178	36.4	71	39.89	—	—
Whether to standardize treatment					4.69	0.030
Yes	136	43.73	32	23.53	—	—
No	175	56.27	61	34.86	—	—
Gravidity					0.55	0.760
1	97	19.84	31	31.96	—	—
2-3	256	52.35	84	32.81	—	—
≥4	136	27.81	49	36.03	—	—
Parity					3.59	0.167
0	195	39.88	72	36.92	—	—
1	205	41.92	59	28.78	—	—
≥2	89	18.20	33	37.08	—	—
Number of children					0.66	0.720
0	207	42.33	73	35.27	—	—
1	206	42.13	65	31.55	—	—
≥2	76	15.54	26	34.21	—	—
Number of spontaneous abortions					1.84	0.399
0	413	84.46	137	33.17	—	—
1	44	9.00	13	29.55	—	—
≥2	32	6.54	14	43.75	—	—
Number of artificial terminations of pregnancy					0.33	0.847
0	276	56.44	90	32.61	—	—
1	118	24.13	42	35.59	—	—
≥2	95	19.43	32	33.68	—	—
Stillbirth					0.01	0.905
0	463	94.68	155	33.48	—	—
1	26	5.32	9	34.62	—	—
Syphilis stage					3.87	0.276
Unknown	109	22.29	29	26.61	—	—
Phase II	4	0.82	2	50.00	—	—
Phase I	21	4.29	6	28.57	—	—
Recessive	355	72.60	127	35.77	—	—
Route of infection					4.77	0.189
Unknown	298	60.94	94	31.54	—	—
Mother-to-child transmission	1	0.20	0	0.00	—	—
Sexual transmission	181	37.01	69	38.12	—	—
Blood transmission	9	1.84	1	11.11	—	—
Husband/partner's current syphilis infection					3.43	0.331
Unknown	207	42.33	69	33.33	—	—
Infected	35	7.16	9	25.71	—	—
Uninfected	102	20.86	30	29.41	—	—
Not detected	145	29.65	56	38.62	—	—
Total	489	100	164	33.54	—	—

RETRACTED

**Table 2:** Logistic regression model analysis of factors related to adverse pregnancy outcomes among syphilis-infected pregnant women.

Factors	*β*	SE	Wald *χ*^2^	*P*	OR (95% CI)
Age	0.034	0.018	3.369	0.066	1.034 (0.998, 1.072)
Titers of first antenatal visit					
<8	—	—	—	—	1.000
>=8	0.825	0.237	12.145	<0.001	2.282 (1.435, 3.631)
Syphilis treatment					
No	—	—	—	—	1.000
Yes	-0.531	0.204	6.788	0.009	0.588 (0.394, 0.877)
Constant	-1.535	0.581	6.991	0.008	0.215

**Table 3:** Unconditional multivariate logistic regression model analysis of adverse pregnancy outcomes in pregnant women treated for syphilis.

Factors	*β*	SE	Wald *χ*^2^	*P*	OR (95% CI)
Age	0.076	0.025	8.842	0.003	1.079 (1.026, 1.134)
Parity	-0.472	0.207	5.173	0.023	0.624 (0.416, 0.937)
Titers of first antenatal visit					
<8	—	—	—	—	1.000
>=8	0.524	0.287	3.334	0.068	1.689 (0.962, 2.965)
Whether to standardize treatment					
No	—	—	—	—	1.000
Yes	-0.628	0.270	5.400	0.020	0.534 (0.314, 0.906)
Constant	-2.142	0.742	8.332	0.004	0.117

**Table 4:** Unconditional multivariate logistic regression model analysis of adverse pregnancy outcomes in pregnant women without treatment for syphilis.

Factors	*β*	SE	Wald *χ*^2^	*P*	OR (95% CI)
Marital status					
First marriage	—	—	—	—	1.000
The other	0.873	0.425	4.224	0.040	2.395 (1.041, 5.508)
Titers of first antenatal visit					
<8	—	—	—	—	1.000
>=8	1.272	0.497	6.560	0.010	3.568 (1.348, 9.442)
Constant	-0.745	0.183	16.606	<0.001	0.475

**Table 5:** Comparison of results features of pregnant women with syphilis with or without treatment during pregnancy.

	No treatment	One course	Two courses	*χ* ^2^	*P*
Titer changes				59.06	<0.01
-5	1 (0.69)	0 (0)	0 (0)	—	—
-4	0 (0)	0 (0)	1 (0.68)	—	—
-3	2 (1.38)	0 (0)	1 (0.68)	—	—
-2	2 (1.38)	1 (0.86)	5 (3.38)	—	—
-1	8 (5.52)	8 (6.90)	15 (10.14)	—	—
0	115 (79.31)	73 (62.93)	64 (43.24)	—	—
1	11 (7.59)	23 (19.83)	37 (25)	—	—
2	6 (4.14)	9 (7.76)	12 (8.11)	—	—
3	0 (0)	2 (1.72)	7 (4.73)	—	—
4	0 (0)	0 (0)	5 (3.38)	—	—
5	0 (0)	0 (0)	1 (0.68)	—	—
Months when specific antibody turns negative				25.93	0.01
3	7 (9.86)	4 (11.43)	23 (32.39)	—	—
6	21 (29.58)	6 (17.14)	15 (21.13)	—	—
9	13 (18.31)	2 (5.71)	11 (15.49)	—	—
12	17 (23.94)	11 (31.43)	7 (9.86)	—	—
15	6 (8.45)	5 (14.29)	6 (8.45)	—	—
18	6 (8.45)	7 (20.00)	8 (11.27)	—	—
21	1 (1.41)	0 (0)	1 (1.41)	—	—
Months to exclude syphilis infection				25.62	0.01
3	7 (8.14)	4 (8.70)	23 (27.06)	—	—
6	40 (45.45)	19 (41.30)	30 (35.29)	—	—
9	13 (14.77)	2 (4.35)	11 (12.94)	—	—
12	17 (19.32)	10 (21.74)	6 (7.06)	—	—
15	4 (4.55)	4 (8.70)	6 (7.06)	—	—
18	6 (6.82)	7 (15.22)	8 (9.41)	—	—
21	1 (1.14)	0 (0)	1 (1.18)	—	—

Note: The results are represented by *n* (%), and the comparison of differences between groups is analyzed by chi-square test. The titer change is the logarithm to the base 2, subtracting that before delivery from that in first test.

**Table 6:** Comparison of results features of one course of treatment at different stages of pregnancy.

	First trimester	Second trimester	Third trimester	*χ* ^2^	*P*
Titer changes				—	0.06
-5	0 (0)	0 (0)	0 (0)	—	—
-4	0 (0)	1 (0.91)	0 (0)	—	—
-3	0 (0)	1 (0.91)	0 (0)	—	—
-2	2 (2.67)	3 (2.73)	1 (1.27)	—	—
-1	8 (10.67)	9 (8.18)	6 (7.59)	—	—
0	37 (49.33)	46 (41.82)	54 (68.35)	—	—
1	17 (22.67)	31 (28.18)	12 (15.19)	—	—
2	5 (6.67)	12 (10.91)	4 (5.06)	—	—
3	2 (2.67)	6 (5.45)	1 (1.27)	—	—
4	4 (5.33)	0 (0)	1 (1.27)	—	—
5	0 (0)	1 (0.91)	0 (0)	—	—
Months when specific antibody turns negative				17.20	0.14
3	12 (29.27)	12 (24.49)	3 (18.75)	—	—
6	10 (24.39)	9 (18.37)	2 (12.50)	—	—
9	6 (14.63)	6 (12.24)	1 (6.25)	—	—
12	8 (19.51)	5 (10.20)	5 (31.25)	—	—
15	2 (4.88)	9 (18.37)	0 (0)	—	—
18	3 (7.32)	7 (14.29)	5 (31.25)	—	—
21	0 (0)	1 (2.04)	0 (0)	—	—
Months to exclude syphilis infection				17.42	0.13
3	12 (23.53)	12 (20.34)	3 (14.29)	—	—
6	20 (39.22)	22 (37.29)	7 (33.33)	—	—
9	6 (11.76)	6 (10.17)	1 (4.76)	—	—
12	8 (15.69)	3 (5.08)	5 (23.81)	—	—
15	2 (3.92)	8 (13.56)	0 (0)	—	—
18	3 (5.88)	7 (11.86)	5 (23.81)	—	—
21	0 (0)	1 (1.69)	0 (0)	—	—

Note: The results are represented by *n* (%), and the comparison of differences between groups is analyzed by chi-square test. The titer change is the logarithm to the base 2, subtracting that before delivery from that in first test. Comparison of titer changes is analyzed by fisher test.

RETRACTED

**Table 7:** Comparison of results features of two courses of treatment at different stages of pregnancy.

	First trimester + first trimester	First trimester + second trimester	First trimester + third trimester	Second trimester + second trimester	Second trimester + third trimester	Third trimester + third trimester	*χ* ^2^	*P*
Titer changes							36.4	0.82
-4	0 (0)	0 (0)	0 (0)	0 (0)	1 (1.47)	0 (0)	—	—
-3	0 (0)	0 (0)	0 (0)	0 (0)	1 (1.47)	0 (0)	—	—
-2	0 (0)	0 (0)	2 (4.76)	1 (7.69)	2 (2.94)	0 (0)	—	—
-1	0 (0)	1 (7.69)	7 (16.67)	1 (7.69)	5 (7.35)	1 (12.50)	—	—
0	2 (66.67)	6 (46.15)	18 (42.86)	4 (30.77)	30 (44.12)	3 (37.50)	—	—
1	0 (0)	2 15.38)	11 (26.19)	5 (38.46)	17 (25.00)	2 (25.00)	—	—
2	0 (0)	2 (15.38)	2 (4.76)	0 (0)	7 (10.29)	1 (12.50)	—	—
3	1 (33.33)	0 (0)	0 (0)	2 (15.38)	4 (5.88)	0 (0)	—	—
4	0 (0)	2 (15.38)	2 (4.76)	0 (0)	0 (0)	1 (12.50)	—	—
5	0 (0)	0 (0)	0 (0)	0 (0)	1 (1.47)	0 (0)	—	—
Months when specific antibody turns negative							—	0.86
3	0 (0)	1 (14.29)	10 (41.67)	1 (33.33)	11 (32.35)	0 (0)	—	—
6	0 (0)	2 (28.57)	4 (16.67)	1 (33.33)	7 (20.59)	1 (50.00)	—	—
9	0 (0)	1 (14.29)	4 (16.67)	1 (33.33)	4 (11.76)	0 (0)	—	—
12	0 (0)	2 (28.57)	3 (12.5)	0 (0)	2 (5.88)	0 (0)	—	—
15	0 (0)	0 (0)	1 (4.17)	0 (0)	5 (14.71)	0 (0)	—	—
18	0 (0)	1 (14.29)	2 (8.33)	0 (0)	4 (11.76)	1 (50.00)	—	—
21	0 (0)	0 (0)	0 (0)	0 (0)	1 (2.94)	0 (0)	—	—
Months to exclude syphilis infection							19.46	0.93
3	0 (0)	1 (11.11)	10 (37.04)	1 (33.33)	11 (35.48)	0 (0)	—	—
6	1 (100.00)	4 (44.44)	7 (25.93)	1 (33.33)	15 (48.38)	2 (66.67)	—	—
9	0 (0)	1 (11.11)	4 (14.81)	1 (33.33)	4 (12.90)	0 (0)	—	—
12	0 (0)	2 (22.22)	3 (11.11)	0 (0)	1 (3.23)	0 (0)	—	—
15	0 (0)	0 (0)	1 (3.70)	0 (0)	5 (16.13)	0 (0)	—	—
18	0 (0)	1 (11.11)	2 (7.41)	0 (0)	4 (12.90)	1 (33.33)	—	—
21	0 (0)	0 (0)	0 (0)	0 (0)	1 (3.23)	0 (0)	—	—

Note: The results are represented by *n* (%), and the comparison of differences between groups is analyzed by chi-square test. The titer change is the logarithm to the base 2, subtracting that before delivery from that in first test. Comparison of titer changes is analyzed by fisher test.

RETRACTED

**Table 8:** Comparison of results features with or without treatment of pregnant women with syphilis with fixed serological titers during pregnancy.

	No treatment	One course	Two courses	*χ* ^2^	*P*
Months when specific antibody turns negative				10.96	0.36
3	3 (7.89)	2 (11.11)	9 (30.00)	—	—
6	11 (28.95)	5 (27.78)	7 (23.33)	—	—
9	7 (18.42)	1 (5.56)	5 (16.67)	—	—
12	8 (21.05)	5 (27.78)	4 (13.33)	—	—
15	5 (13.16)	1 (5.56)	2 (6.67)	—	—
18	4 (10.53)	4 (22.22)	3 (10.00)	—	—
Months to exclude syphilis infection				14.76	0.14
3	3 (6.00)	2 (10.53)	9 (28.13)	—	—
6	25 (50.00)	6 (31.58)	10 (31.25)	—	—
9	7 (14.00)	1 (5.26)	5 (15.63)	—	—
12	8 (16.00)	5 (26.32)	3 (9.37)	—	—
15	3 (6.00)	1 (5.26)	2 (6.25)	—	—
18	4 (8.00)	4 (21.05)	3 (9.37)	—	—

Note: The serologically fixed pregnant women are those whose first titer and pre-delivery titer remain unchanged, and both are less than 1 : 8. The results are represented by *n* (%), and the comparison of differences between groups is analyzed by chi-square test.

**Table 9:** Comparison of results features of pregnant women with syphilis with or without treatment during pregnancy between high titer group and low titer group.

	High titer group			Low titer group			*χ* ^2^	*P*
	No treatment	One course	Two courses	No treatment	One course	Two courses		
Titer changes							164.16	<0.01
-5	0 (0)	0 (0)	0 (0)	1 (0.81)	0 (0)	0 (0)	—	—
-4	0 (0)	0 (0)	0 (0)	0 (0)	0 (0)	1 (0.94)	—	—
-3	0 (0)	0 (0)	0 (0)	2 (1.61)	0 (0)	1 (0.94)	—	—
-2	1 (4.76)	0 (0)	0 (0)	1 (0.81)	1 (1.25)	5 (4.72)	—	—
-1	0 (0)	2 (5.56)	3 (7.14)	8 (6.45)	6 (7.50)	12 (11.32)	—	—
0	18 (85.71)	19 (52.78)	10 (23.81)	97 (78.23)	54 (67.50)	54 (50.94)	—	—
1	1 (4.76)	7 (19.44)	11 (26.19)	10 (8.06)	16 (20.00)	26 (24.53)	—	—
2	1 (4.76)	6 (16.67)	5 (11.90)	5 (4.03)	3 (3.75)	7 (6.60)	—	—
3	0 (0)	2 (5.56)	7 (16.67)	0 (0)	0 (0)	0 (0)	—	—
4	0 (0)	0 (0)	5 (11.90)	0 (0)	0 (0)	0 (0)	—	—
5	0 (0)	0 (0)	1 (2.38)	0 (0)	0 (0)	0 (0)	—	—
Months when specific antibody turns negative							34.68	0.25
3	0 (0)	0 (0)	4 (23.53)	7 (10.61)	4 (14.29)	19 (35.85)	—	—
6	2 (50.00)	0 (0)	5 (29.41)	19 (28.79)	6 (21.43)	10 (18.87)	—	—
9	0 (0)	1 (14.29)	3 (17.65)	13 (19.70)	1 (3.57)	8 (15.09)	—	—
12	1 (25.00)	3 (42.86)	2 (11.76)	16 (24.24)	8 (28.57)	5 (9.43)	—	—
15	0 (0)	1 (14.29)	1 (5.88)	6 (9.09)	4 (14.29)	5 (9.43)	—	—
18	1 (25.00)	2 (28.57)	2 (11.76)	5 (7.58)	5 (17.86)	6 (11.32)	—	—
21	0 (0)	0 (0)	0 (0)	1 (1.52)	0 (0)	1 (1.89)	—	—
Months to exclude syphilis infection							32.96	0.32
3	0 (0)	0 (0)	4 (21.05)	7 (8.33)	4 (11.43)	19 (28.79)	—	—
6	2 (50.00)	5 (45.45)	7 (36.84)	38 (45.24)	14 (40.00)	23 (34.85)	—	—
9	0 (0)	1 (9.09)	3 (15.79)	13 (15.48)	1 (2.86)	8 (12.12)	—	—
12	1 (25.00)	3 (27.27)	2 (10.53)	16 (19.05)	7 (20.00)	4 (6.06)	—	—
15	0 (0)	0 (0)	1 (5.26)	4 (4.76)	4 (11.43)	5 (7.58)	—	—
18	1 (25.00)	2 (18.18)	2 (10.53)	5 (5.95)	5 (14.29)	6 (9.09)	—	—
21	0 (0)	0 (0)	0 (0)	1 (0.65)	0 (0)	1 (1.52)	—	—

Note: The results are represented by *n* (%), and the comparison of differences between groups is analyzed by chi-square test. The titer change is the logarithm to the base 2, subtracting that before delivery from that in first test.

RETRACTED

## Data Availability

The data in this study are all derived from the information system. As it involves the privacy of pregnant women with syphilis and their children, the data cannot be fully disclosed. If the research colleagues are interested in this, you can contact the corresponding author via email to obtain the data.
